# Assessment of the Potential Health Risk of Gold Nanoparticles Used in Nanomedicine

**DOI:** 10.1155/2022/4685642

**Published:** 2022-07-29

**Authors:** Monika Dvorakova, Lubomir Kuracka, Ingrid Zitnanova, Sona Scsukova, Jozef Kollar, Katarina Konarikova, Lucia Laubertova

**Affiliations:** ^1^Department of Medical Chemistry, Biochemistry and Clinical Biochemistry, Faculty of Medicine, Comenius University, Sasinkova 2, 813 72 Bratislava, Slovakia; ^2^Institute of Experimental Endocrinology, Biomedical Research Center, Slovak Academy of Sciences, Dubravska cesta 9, 845 05 Bratislava, Slovakia; ^3^Polymer Institute, Slovak Academy of Sciences, Dubravska cesta 9, 845 05 Bratislava, Slovakia

## Abstract

Due to unique properties, nanoparticles (NPs) have become a preferred material in biomedicine. The benefits of their use are indisputable, but their safety and potential toxicity are becoming more and more important. Especially, excessive production of reactive oxygen species (ROS) induced by the strong oxidation potential of metal NPs could evoke adverse effects associated with damage to nucleic acids, proteins and lipids. Our study gives a view on the potential cytotoxicity of gold NPs (Au NPs) of different size from the perspective of the redox state of healthy (HEK 293 T) and cancer (A375 and A594) cell lines. These cells were incubated in the presence of two concentrations of Au NPs for 24 h or 72 h and total antioxidant capacity, 8-isoprostane, and protein carbonyl levels were determined. Furthermore, the activity of antioxidant enzymes such as superoxide dismutase, glutathione peroxidase, and catalase was detected in cell lysates. Our results compared to the results of other laboratories are very contradictory. The outcomes also differ between healthy and cancer cell lines. However, there are certainly changes in the activities of antioxidant enzymes, as well as the damage to biological molecules due to increased NP-induced oxidative stress. But the final decision of the effect of Au NPs on the oxidative state of selected cell lines requires further research.

## 1. Introduction

Nanoparticles (NPs) are defined as materials up to 100 nm in size. Their large surface/volume ratio together with the surface treatment gives them unique characteristics, thus improving their mechanical and catalytic properties. Last, but not least, they have the ability to absorb high amounts of drugs, e.g., in cancer treatment. In addition, they are able to pass blood-brain barrier (BBB) that enormously increases their potential for pharmacological use [1, 2].

One of the consequences of NP overuse in all areas of industry and medicine is an increased interest of scientists in side effects of their application. This topic can be very delicate, especially in the field of biomedicine, where the overuse of NPs can influence the healthy life of individuals.

After the NP enters the body, it is distributed to the organs and tissues via the bloodstream. Quantitative analysis results from *in vivo* studies on rodents showed that accumulation of NPs varied in different tissues (liver, spleen, kidney, and lung) depending on a route of NP administration (intravenous, subcutaneous, oral, and inhalation). Often by targeted transport and the transport through the BBB, and over various mechanisms, NPs can react with biological components and cause numerous adverse effects. One of the possible mechanisms of this destructive consequence may be the formation of oxidative stress associated with a damage to biologically important molecules, such as nucleic acids [3], proteins [4], or lipids [5]. In addition, the activities of antioxidant enzymes can be affected leading to the change in the redox state of the organism [6, 7].

Metal NPs, especially noble metal NPs, form a special group of NPs with an application in medicine. The surface of these materials can be modified in many ways with several chemical functional groups which enable them to conjugate with for example ligands, antibodies, or drugs [8, 9]. Depending on the treatment of NPs surface, their properties also unfold. Metal NPs, e.g., gold NPs (Au NPs), together with their surface modification, create opportunities for use in photothermal therapy, cancer cell detection, gene regulation, or imaging techniques [10]. In particular, Au NPs play an important role in cancer imaging, pathogenesis, and disease progression with their ability to cross the cell nucleus [11, 12]. Targeting of NPs to for example cancer cells can be achieved by binding a suitable ligand to NPs surface. These systems are very specific, including the binding a huge number of therapeutics/diagnostics. In addition, controlling the size of the NPs allows them to avoid the body's immune system reaction and thus stay in the bloodstream longer. All of these facts guarantee the delivery of the NPs to targeted cell [13]. In biomedicine, in addition to the declared purposes, Au NPs modified by bound ligands or activated by photothermal therapy have one of the most significant antibacterial effects among noble metal NPs [14, 15].

Even though the pros of using NPs in medicine are undeniable, some adverse effects have also been reported. Diverse NPs can cause different harmful effects depending on their size and type [16–19]. They can cause toxicity on the molecular (conformation changes, aggregation of molecules, and loss of function), cellular (reactive oxygen species (ROS) formation and compartment disruption), or tissue levels (inflammation, damage) [20–22]. Especially, the formation of ROS belongs to the most studied mechanisms of the NPs toxicity [17, 19]. Furthermore, NPs could interfere with antioxidant enzyme genes such as *sod1* or *gpx1* and thus influence the redox state of the cell [6, 7].

Oxidative stress (redox imbalance) can be briefly defined as an imbalance between oxidants and antioxidants in favor of oxidants [23]. Antioxidants represent the defense of organism against harmful effects of oxidants. They include mainly endogenous high molecular weight antioxidant enzymes and exogenous low molecular weight compounds [24]. Reactive oxygen (nitrogen) species (RO(N) S) seem to be crucial in the development of oxidative stress. They can be either radicals (with an unpaired electron) (hydroxyl radical, superoxide, and nitric oxide) or non-radicals (hydrogen peroxide, ozone, singlet oxygen, and peroxynitrite). Their elevated concentration together with depletion of antioxidants can lead to oxidative stress establishment. This redox imbalance can modify nucleic acids, proteins and lipids [25]. If not controlled, oxidative stress can speed up ageing and be the one of reasons of many diseases (e.g., cancer, cardiovascular diseases, atherosclerosis, diabetes mellitus, neurological diseases, rheumatoid arthritis, and preeclampsia) [25–28]. However, in higher organisms, NO can be involved as a signal molecule (regulation of vascular tone and signal transduction from membrane receptors). In addition, at physiological conditions, ROS are produced, e.g., as a side product of respiratory chain, or by phagocytic NADPH oxidase, cyclooxygenase, or lymphocytes [26]. Thus, the effects of RO(N) S re not only harmful, but they contribute to the precise functioning of the organism.

Various types of NPs (e.g., TiO_2_, ZnO, SiO_2_, Au, and Ag NPs) are known to be very reactive with hydrogen peroxide to form ROS via the Haber-Weiss or Fenton reactions [29, 30]. Hydroxyl radical formed in these reactions is very reactive and toxic, reacting with DNA, proteins, and lipids [31], and together with the superoxide radical, its formation can lead to irreversible modulations of many intracellular pathways [32, 33]. Also, e.g., ZnO NPs under the UV radiation cause the depletion of reduced glutathione via the hydroxyl radical and hydrogen peroxide formation [34]. Thus, ROS are responsible for the toxicity of NPs due to oxidative stress [32]. Nevertheless, not all NPs can cause the oxidative stress. This effect depends on their physical and chemical properties (solubility, adsorption, and crystalline phase). Consequently, the size of the NPs is not the limiting factor to induce oxidative stress and harmful side effects [35].

Due to their huge potential in diagnosis and treatment of diseases, nanotechnology appears to have an irreplaceable role in biomedicine [36]. Nowadays, the question, whether the benefits of NP use outweigh the risks, is the subject of research. Especially in biomedicine, the safety of NPs is one of the most important aspects.

Despite the fact that NPs research is advancing at an enormous pace, there is a lack of information on the consequences of using Au NPs on the induction of oxidative stress. The objective of this work was to determine the effect of Au NPs of different sizes (20 and 100 nm) and different concentrations on parameters of the redox status, such as the total antioxidant status, lipid and protein oxidation markers, and antioxidant enzyme activities (glutathione peroxidase (GPx), superoxide dismutase (SOD), and catalase) in selected healthy and cancer cell lines derived from different tissues.

## 2. Materials and Methods

### 2.1. Gold Nanoparticles

Gold nanoparticles (Au NPs) of 20 and 100 nm (catalog nos. 753610 and 753688, respectively; both gold colloid, OD 1, stabilized suspension in 0.1 mM phosphate buffered saline (PBS), and reactant-free) were purchased from Sigma-Aldrich (Merck KGaA, Darmstadt, Germany). Dynamic light scattering (DLS) analysis (Malvern Instrument Zetasizer Nano, UK) of Au NP suspensions showed one peak with hydrodynamic size 20.93 ± 4.82nm for 20nm Au NPs and 76.27 ± 20.74 nm for 100 nm Au NPs. Polydispersity index (PDI) of Au NP suspension was 0.156 and 0.054 for 20 and 100 nm NPs, respectively.

The concentration of stock NP suspension was ~6.54 × 10^11^ particles (pcs)/mL for 20 nm Au NPs and ~3.8 × 10^9^ pcs/mL for 100 nm Au NPs. Before dilution with the cell culture medium to achieve the final assay concentration, the stock NP suspension was sonicated for 5 min in ultrasound water bath cooled with ice. The NP dilutions were mixed again by vortex to disperse the NPs as homogenously as possible before adding the tested NPs to the cell cultures.

### 2.2. Cell Cultures

Human melanoma A375 cells, lung cancer A549 cells, and healthy embryonic kidney HEK 293 T cells were purchased from American Type Culture Collection (ATCC), Rockville, MD, USA. All cell lines were cultured in the complete Dulbecco's Modified Eagle's Medium supplemented with 10% (vol./vol.) heat-inactivated fetal bovine serum, penicillin (100 U/mL), and streptomycin (100*μ*g/mL). All cell lines were grown at 37 °C in humidified 5% CO_2_ and 95% air atmosphere. For our experiments, a cell inoculum of 2 × 10^4^ cells/mL for the HEK 293 T cell line was used and of 1 × 10^5^ cells/mL for A375 and A549 cell lines was used. All cell lines were incubated for 24 h or 72 h prior to analyzing the selected parameters.

### 2.3. Cell Proliferation

Proliferation of cells was determined by 3-(4,5-dimethylthiazol-2-yl)-2,5-diphenyltetrazolium bromide (MTT) assay in 96-well plate [37]. The effect of Au NPs on proliferation of cells cultured for 24 h or 72 h was expressed as % of viability relative to the untreated control cells of the tested cell line. All experiments were repeated at least three times.

### 2.4. Gold Nanoparticle Treatment

To the adherent cell lines A375, A549, and HEK 293 T Au NPs were added: Au NPs of 20 nm at a final concentration of 1.6 × 10^9^ pcs/mL; 1.6 × 10^11^ pcs/mL of culture medium and Au NPs of 100 nm at a final concentration of 1.6 × 10^7^; and 1.6 × 10^9^ pcs/mL of culture medium. Cells were cultured with Au NPs for 24 h or 72 h.

The adherent cell lines HEK 293 T, A375, and A549 were cultured with two different concentrations of Au NPs: 1.6 × 10^9^ pcs/mL and 1.6 × 10^11^ pcs/mL for 20 nm Au NPs and 1.6 × 10^7^ and 1.6 × 10^9^ pcs/mL for 100 nm Au NPs for 24 h and 72 h.

After the 24 h and 72 h treatment with/without NPs, the medium was aspirated, and cells were washed three times in PBS. Cell lysates were prepared using lysis RIPA buffer and sonification with three 5 s on/off cycles at 50% power at 4 °C (Kraintek 10, Slovakia). Lysates were collected and cleared by centrifugation, aliquoted and frozen (at −80 °C) for further analysis.

### 2.5. Protein Concentration

Protein concentration in tested cell lysates was measured using a Pierce™ BCA Protein Assay kit (Thermo Scientific, USA). The concentration was expressed in mg/mL.

Since the concentration of proteins in lysates reflects the number of cells which were lysed and examined, all the parameters determined were related to the amount of proteins.

### 2.6. Trolox Equivalent Antioxidant Capacity (TEAC)

Spectrophotometric method [38] was used for screening of antioxidant capacity in cell lysates. As a standard, trolox (water-soluble analogue of vitamin E) was used. TEAC values were expressed in mmol of trolox/*μ*g of proteins.

### 2.7. 8-Isoprostane

The concentration of 8-isoprostane was determined in all three cell lines using an 8-isoprostane ELISA kit (Cayman Chemical, USA). The concentration was calculated in pg/mL.

### 2.8. Protein Carbonyls

To evaluate protein carbonyl levels, the commercial kit OxiSelect™ Protein Carbonyl ELISA Kit (Cell Biolabs, Inc., USA) was used. Protein carbonyl concentrations were expressed in nmol/mg of proteins.

### 2.9. Superoxide Dismutase Activity

To evaluate SOD activity in cell lysates, SOD Assay Kit (Sigma-Aldrich Co., USA) was used. Enzyme activity was expressed as inhibition rate percent, where 1 U of SOD activity was defined as the amount of enzyme able to inhibit the rate of chromagen reduction by 50%.

### 2.10. Glutathione Peroxidase Activity

GPx activity was determined in cell lysates using the commercial Glutathione Peroxidase Assay Kit (Cayman Chemical, USA). Activity of the enzyme was expressed in U/mg of proteins.

### 2.11. Catalase Activity

To measure the catalase (Cat) activity in cell lysates, the Catalase Assay kit (Cayman, USA) was used. The activity was expressed in U/mg of proteins.

### 2.12. Statistical Analysis

We analyzed the data of cell proliferation using Two-way ANOVA test with Dunnett multiple comparison and the mean ± standard error of the mean (SEM) was used. Due to the not normally distributed data of other parameters, we analyzed the data using nonparametric Kruskal-Wallis test. The median with interquartile range (IQR) with upper and lower quartile values was used. All experiments were repeated three times. We performed statistical tests using the statistical program IBM SPSS Statistic 22 and StatsDirect® 3.2.8 (Stats Direct Sales, Sale, Cheshire M33 3UY, UK). The significance level was defined as *P* < 0.05.

## 3. Results

### 3.1. Cell Proliferation

In primary screening, the effect of different sizes of Au NPs (20 and 100 nm) and their different concentrations on cell proliferation were investigated during 24 h and 72 h. Incubation of A549, A375, and HEK 293 T cells with different concentrations of 20 nm Au NPs for 24 h and 72 h had no significant effect on cell proliferation compared to untreated control cells (Figures 1(a), 1(b), and 1(c)).

After 24 h and 72-h incubation of A549, A375, and HEK 293 T cells with 100 nm Au NPs, only the highest concentration of 100 nm Au NPs (1.6×10^9^ pcs/mL) significantly decreased (*P* < 0.05 and *P* < 0.01) proliferation of cells by 40-50% in comparison to untreated control cells. Lower concentrations of 100 nm Au NPs used had no significant effect on cell proliferation of A549, A375, and HEK 293 T cells.

### 3.2. HEK 293 T Cell Line

#### 3.2.1. Trolox Equivalent Antioxidant Capacity (TEAC)

In healthy HEK 293 T cells, we found no change in TEAC of cells incubated with selected concentrations of Au NPs (Table 1).

#### 3.2.2. 8-Isoprostane

A 24-hour incubation of HEK 293 T cells with Au-NPs (20 nm and 100 nm) had no effect on the level of the marker of lipid oxidation-8-isoprostane in comparison to control cells and different NPs concentrations as well (Table 2).

Interesting is the finding of elevated 8-isoprostane levels in control cells after 72-h incubation (compared to 24 h, *P* < 0.05). Similarly, their concentration increased over time also in case of incubation of cells with 100 nm Au NPs at both concentrations used (*P* < 0.05). In cells incubated with 20 nm NPs, no change in 8-isoprostane concentrations over time was recorded (Table 2).

Incubation of HEK 293 T cells with 20 nm NPs significantly reduced the 8-isoprostane levels at higher NPs concentration: 1.6 × 10^11^ pcs/mL after 72 h compared to control (*P* < 0.001). However, 100 nm NPs showed no effect on 8-isoprostane level when compared to control cells.

Similarly, the concentration of 8-isoprostane increased over time when cells were incubated with 100 nm Au NPs at both concentrations used (Table 2).

#### 3.2.3. Protein Carbonyls

After 24-h incubation of HEK 293 T cells with Au NPs, no effect of 20 nm Au NPs on the production of protein carbonyls was determined (Table 3). Compared to control cells, concentration of protein carbonyls was decreased significantly when 100 nm NPs were used at a concentration of 1.6 × 10^9^ pcs/mL (*P* < 0.05). In addition, with elevated concentration of NPs of 20 nm size, the level of protein carbonyls decreased significantly (*P* < 0.05).

After 72-h incubation of control cells, the concentration of protein carbonyls increased significantly compared to 24-h incubation (*P* < 0.01). Au NPs of 100 nm at the concentration of 1.6 × 10^9^ pcs/mL significantly reduced the level of protein carbonyls compared to this control (*P* < 0.01) (Table 3).

### 3.3. Superoxide Dismutase (SOD) Activity

Au NPs of 20 and 100 nm at the tested concentrations had no effect on SOD activity of HEK 293 T cells for both time intervals compared to control cells (Table 4).

When we compared SOD activity of HEK 293 T cells incubated for 24 h and 72 h with 100 nm Au NPs at the concentration of 1.6 × 10^9^ pcs/mL, we found the decrease of activity over time (*P* < 0.05) (Table 4).

### 3.4. Glutathione Peroxidase (GPx) Activity

Incubation of healthy HEK 293 T cells with both sizes of Au NPs for 24 h or 72 h showed no significant changes in the GPx activity (Table 5).

### 3.5. Catalase Activity

Compared to control cells, 20 nm Au-NPs (1.6 × 10^11^ pcs/mL) as well as 100 nm Au NPs (1.6 × 10^7^ pcs/mL) after 24-h incubation with cells significantly increased catalase activity in HEK 293 T cells after 24-hour incubation (*P* < 0.05) (Table 6).

Compared to 24-h incubation, a 72-hour incubation of 20 nm Au NPs with HEK 293 T cells significantly increased catalase activity at the NPs concentration of 1.6 × 10^9^ pcs/mL (*P* < 0.05) (Table 6).

### 3.6. Cell Line A375

#### 3.6.1. Total Antioxidant Capacity (TEAC)

After 24-h incubation of A375 cells with either 20 nm or 100 nm Au NPs, we found no significant differences between control and cells incubated with the NPs (Table 7).

On the contrary, when we compared TEAC after 72-h incubation, in case of incubation of A375 cells with 100 nm NPs at the concentration of 1.6 × 10^7^ pcs/mL, we found a decrease of TEAC compared to control (*P* < 0.05). In addition, A375 cells incubated with 100 nm NPs at the concentration of 1.6 × 10^7^ pcs/mL showed a lower TEAC compared to NP concentration of 1.6 × 10^9^ pcs/mL (*P* < 0.001) (Table 7).

Interesting was the finding of TEAC significant increase over time (72 h vs. 24-h incubation) after treatment of A375 cells with Au NPs of both sizes (20 and 100 nm) at the concentration of 1.6 × 10^9^ pcs/mL (*P* < 0.01 for 20 nm NPs; *P* < 0.05 for 100 nm NPs) (Table 7).

#### 3.6.2. 8-Isoprostane

After 24-h incubation of A375 cells with 20 nm NPs at the concentration of 1.6 × 10^11^ pcs/mL, we found an increased concentration of 8-isoprostane compared to control cells (*P* < 0.05). On the contrary, elevated concentration (*P* < 0.05) of 8-isoprostane was found also after 72-h incubation of A375 cells with 20 nm NPs at the concentration of 1.6 × 10^9^ pcs/mL compared to control (Table 8).

When we examined the 8-isoprostane concentration in A375 cells over time (24 h vs. 72-h incubation), its concentration was significantly higher (*P* < 0.05) in case of 72-h incubation of cells with 20 nm Au NPs at the concentration of 1.6 × 10^9^ pcs/mL.

Furthermore, 20 nm Au NPs at concentration of 1.6 × 10^11^ pcs/mL induced significantly higher generation of 8-isoprostane in A375 cells compared to lower concentration of NPs (1.6 × 10^9^ pcs/mL) after 24-h incubation (*P* < 0.05) (Table 8).

#### 3.6.3. Protein Carbonyls

Treatment of A375 cells for 24 h and 72 h with Au NPs of 20 nm at both tested concentrations (1.6 × 10^9^ and 1.6 × 10^11^ pcs/mL) did not significantly affect the level of protein carbonyls in cells compared to corresponding controls. Compared to control, the level of protein carbonyls was significantly higher in cells incubated for 24 h with 100 nm Au NPs at concentrations of 1.6 × 10^7^ pcs/mL and 1.6 × 10^9^ pcs/mL (*P* < 0.001) (Table 9).

Over time (24 h vs. 72-h incubation), the concentration of protein carbonyls in control A375 cells was significantly elevated after 72-h incubation (*P* < 0.01). Comparable effect was also demonstrated in A375 cells incubated with 20 nm Au NPs at both tested concentrations (in both cases *P* < 0.05), or after incubation with 100 nm Au NPs at the concentration of 1.6 × 10^7^ pcs/mL (*P* < 0.01) (Table 9).

#### 3.6.4. Superoxide Dismutase (SOD) Activity

Au NPs of both size at all concentrations tested had no effect on SOD activity of A375 cells after 24 h and 72-h incubation (Table 10).

When we track the change of SOD activity over time, cancer A375 cells incubated with 20 nm NPs at the concentration of 1.6 × 10^9^ pcs/mL had elevated enzymatic activity after 72-h incubation compared to 24 h (*P* < 0.05) (Table 10).

#### 3.6.5. Glutathione Peroxidase (GPx) Activity

Incubation of A375 cells for 24 h and 72 h with 20 nm and 100 nm Au-NPs at all concentrations used caused no significant changes in the GPx activity (Table 11).

#### 3.6.6. Catalase Activity

Compared to control cells, after 24-h incubation of A375 cells with 20 nm Au NPs at concentration of 1.6 × 10^11^ pcs/mL, as well as with 100 nm NPs at concentration of 1.6 × 10^7^ pcs/mL, we observed a significantly lower catalase activity (*P* < 0.05) in cells (*P* < 0.01 in case of 20 nm NPs at the concentration of 1.6 × 10^11^ pcs/mL and *P* < 0.05 in case of 100 nm Au NPs with the concentration of 1.6 × 10^7^ pcs/mL). On the contrary, after 72-h incubation of A375 cells with 100 nm Au NPs at the concentration of 1.6 × 10^9^ pcs/mL, the activity of catalase was higher (*P* < 0.001) compared to control cells (Table 12).

Interesting was the finding of reduced enzymatic activity over time (24 h vs 72 h of incubation) found in control, (*P* < 0.01) as well as in A375 cells treated with 20 nm NPs at concentrations of 1.6 × 10^9^ and 1.6 × 10^11^ pcs/mL.

### 3.7. A549 Cell Line

#### 3.7.1. Total Antioxidant Capacity (TEAC)

In case of 24-h incubation of A549 cells, compared to control, we found an increased TEAC in cells incubated with 20 nm Au NPs (1.6 × 10^11^ pcs/mL, *P* < 0.05), as well as in cells incubated with 100 nm Au NPs (1.6 × 10^7^ pcs/mL, *P* < 0.05). Inhibitory effect on TEAC in A549 cells was determined after 72-h incubation of cells with 20 nm Au NPs (1.6 × 10^11^ pcs/mL, *P* < 0.01) and in cells incubated with 100 nm Au NPs (1.6 × 10^7^ pcs/mL, *P* < 0.001) (Table 13).

Comparing TEAC over time (24 h vs. 72-h incubation), longer incubation increased TEAC of control cells and decreased TEAC of cells treated with 20 nm Au NPs at c = 1.6 × 10^11^ pcs/mL (*P* < 0.05) and with 100 nm Au NPs at the concentration of 1.6 × 10^7^ pcs/mL (Table 13).

Incubation of A549 cells with 20 nm Au NPs at higher concentration (1.6 × 10^11^ pcs/mL) induced an increase in TEAC of cells compared to their incubation with 20 nm Au NPs of lower concentration (1.6 × 10^9^ pcs/mL) (*P* < 0.05).

After 24-h incubation, TEAC was significantly higher in A549 cells treated with 100 nm Au NPs at lower concentration (1.6 × 10^7^ pcs/mL), compared to cells incubated with NPs of the same size but the higher concentration (*P* < 0.001). On the contrary, after 72-h incubation, the 100 nm Au NPs at the concentration of 1.6 × 10^7^ pcs/mL induced lower TEAC in A549 cells compared to Au NPs of the same size with the lower concentration (1.6 × 10^9^ pcs/mL) (*P* < 0.05).

#### 3.7.2. 8-Isoprostane

After 24-h incubation of A549 cells with Au NPs with cells, we determined lower 8-isoprostane level in cells treated with 20 nm Au NPs at both concentrations (*P* < 0.01 for 1.6 × 10^9^ pcs/mL and *P* < 0.05 for 1.6 × 10^11^ pcs/mL) compared to control. Similar result, the decrease of 8-isoprostane concentration was found after 72-h incubation of A549 cells with 100 nm Au NPs at higher concentration (1.6 × 10^9^ pcs/mL) (*P* < 0.05) (Table 14).

When we compared the 8-isoprostane concentration over time, its level was significantly increased after 72-h incubation of A549 cells with 20 nm Au NPs of 1.6 × 10^11^ pcs/mL concentration (*P* < 0.01) and 100 nm Au NPs at the concentration of 1.6 × 10^7^ pcs/mL (*P* < 0.01) (Table 14).

Interestingly, when we compared 8-isoprostane concentration in A549 cells incubated with 100 nm Au NPs for 72 h, its concentration was lower in cells treated with higher concentration of NPs (1.6 × 10^7^ pcs/mL vs. 1.6 × 10^9^ pcs/mL) (*P* < 0.01) (Table 14).

#### 3.7.3. Protein Carbonyls

Compared to 24-h incubation, 72-h incubation of A549 control cells caused a significant increase in protein carbonyls level (*P* < 0.01) (Table 15).

Incubation of A549 cells with 20 nm Au NPs induced a time-dependent elevation of protein carbonyls concentration (*P* < 0.01) at both concentrations of NPs. The same effect was found in cells incubated with 100 nm Au NPs of both tested concentrations (*P* < 0.05).

It was interesting to find the rise of protein carbonyls level with the increased concentration of Au NPs of both sizes (for 20 nm NPs after 24-h incubation *P* < 0.001 and for 100 nm NPs after 72-h incubation *P* < 0.01).

#### 3.7.4. Superoxide Dismutase (SOD) Activity

Treatment of cancer A549 cells with Au NPs of both sizes (20 and 100 nm) at concentrations tested had no significant effect on SOD activity compared to control cells (Table 16).

Only the 72-h incubation of cancer A549 cells with 20 nm Au NPs of 1.6 × 10^9^ pcs/mL concentration caused a significant elevation in SOD activity compared to 24-h incubation of cells with NPs of the same size and concentration (*P* < 0.05) (Table 16).

#### 3.7.5. Glutathione Peroxidase (GPx) Activity

Incubation of cancer A549 cells with 20 nm and 100 nm Au NPs caused no significant changes in the GPx activity compared to control cells (Table 17).

In case of control cells, their 72-h incubation decreased GPx activity significantly compared to 24-h incubation (*P* < 0.05) (Table 17).

#### 3.7.6. Catalase Activity

Treatment of cancer A549 cells with Au NPs of both sizes for 24 h did not significantly affect catalase activity of cells compared to controls. A549 cells incubated with 20 nm and 100 nm Au NPs at higher tested concentrations (1.6 × 10^11^ pcs/mL and 1.6 × 10^9^ pcs/mL) for 72 h had significantly increased catalase activity (in both cases *P* < 0.001) compared to controls (Table 18).

If we relate catalase activities after 24 h vs. 72 h incubation of cells with NPs, 100 nm Au NPs (1.6 × 10^9^ pcs/mL) induced elevation of enzymatic activity of A549 cells after 72 h (*P* < 0.01) (Table 18).

At both incubation times, A549 cells incubated with 20 nm Au NPs (1.6 × 10^11^ pcs/mL) had increased catalase activity compared to cells incubated with NPs of the same size, but lower concentration (1.6 × 10^9^ pcs/mL) (for 24 h *P* < 0.001 and for 72 h *P* < 0.01) (Table 18).

Similarly, when we examine the effect of 100 nm Au NPs (concentration of 1.6 × 10^9^ pcs/mL) on the catalase activity of A549 cells treated for 72 h, we found increased catalase activity compared to cells treated for 24 h with Au NPs of the same size and concentration (*P* < 0.05).

## 4. Discussion

The size of NPs is considered one of the crucial, although not the only factor responsible for the NPs toxicity [39–42]. It means, the smaller NP, the higher association with its toxic effect. In our study, we assessed the effects of two different sizes of NPs, 20 nm and 100 nm, of different concentrations with regard to different incubation times (24 and 72 h) with different cell lines—healthy embryonic kidney cells (HEK 293 T) and human melanoma (A375) and lung (A549) cancer cell lines. Total antioxidant capacity (TEAC), 8-isoprostane, and protein carbonyl levels, as well as the activities of antioxidant enzymes, glutathione peroxidase (GPx), superoxide dismutase (SOD), and catalase, were determined.

NPs are known to decrease the viability of healthy and cancer cell lines, including HEK 293 cells [41, 43, 44]. In spite of it, our results indicate that except of the 100 nm NPs with the concentration of 1.6 × 10^9^ pcs/mL, both selected sizes and concentrations of NPs had no effects on the viability of any cells used in this study.

NPs can act as artificial redox systems by mimicking various antioxidants and targeting selected tissues which may reduce the RO(N) S induced damage to biomolecules [45]. Numerous studies confirmed antioxidant activity of metal NPs [46–48]. For example, Keshari et al. [49] found a higher antioxidant activity of silver (Ag) NPs measured by 2,2-diphenyl-1-picryl-hydrazyl-hydrate (DPPH) method, as well as their higher hydroxyl radical scavenging activity compared to vitamin C. Likewise, Annu et al. [50] also indicated that treatment of A549 cells with Ag NPs resulted in the reduction of ROS formation, suggesting a higher antioxidant capacity of NPs. Confirmed antioxidant activity of these metal NPs is in agreement with our findings of increased antioxidant activity (measured by TEAC) of healthy HEK 293 T cells treated with 100 nm Au NPs (1.6 × 10^9^ pcs/mL) after 72-h incubation compared to untreated cells. Similar results were obtained in cancer cell line A549 already after 24-h incubation with 20 nm Au NPs (1.6 × 10^11^ pcs/mL), as well as with 100 nm NPs (1.6 × 10^7^ pcs/mL). On the contrary, the 72-h incubation of cells with both sizes of Au NPs caused the decrease in antioxidant capacity of A549 and A375 cells compared to controls.

It is known that NPs of various types and sizes can among others enter the mitochondria, which play an important role in the formation of free radicals [51]. Thus, they can modify their production and affect the activity of enzymes involved in the antioxidant defense of the cell [52]. Different studies reported different effects of metal NPs on enzymatic activities. According to Siddiqi [53], treatment of rats with 20 nm Au NPs (dose 20 *μ*g/kg body weight, concentration of 0.01%) caused no significant change in activity of SOD in tissues excluding kidneys, where the activity was elevated. However, in our case, the treatment of kidney HEK 293 T cells with 100 nm Au NPs (1.6 × 10^9^ pcs/mL) for 72 h decreased the SOD activity compared to 24-h incubation. On the other hand, if 20 nm NPs (1.6 × 10^9^ pcs/mL) were incubated with cancer cell lines (A375 and A549), the SOD activity increased compared to 24-h incubation. Whether the different behavior of healthy and cancer cells incubated with Au NPs is caused by a higher imbalance between oxidants and antioxidants in cancer cells or by the ability of Au NPs to activate SOD should be the goal of further research. On the other hand, despite a confirmed higher mimetic GPx activity of gold@platinum NPs (Au: Pt ratio was 4 : 1, Au NPs of size 90 × 40 nm (length x diameter), and Pt NPs size 3 nm in diameter) compared to mimetic ascorbic acid antioxidant activity [54], in our samples with Au NPs, the activity of GPx remained unchanged in all cell lines at all concentrations. Our results are in sync with the research of Canli and Canli [55] who found no effects of metal oxide (Al_2_O_3_, CuO, and TiO_2_) NPs on the cell GPx activity, but, on the contrary, decreased activity of SOD in the liver tissue of Nile fish compared to unexposed fish. Catalase activity according to their results was also reduced, but our research suggested increased catalase activity with time and concentration of NPs in cancer cell lines. Another study [56] examined the effect of Pt NPs on A549 cells and determined the elevation of SOD, GPx, as well as catalase activities. Their results indicate that Pt NPs might be a promising agent in the treatment of lung cancer. These data are also consistent with our results. We found a similar increase of SOD and catalase activities in cancer cell lines (but no effect on GPx activity). All of these findings confirm the possible antioxidative properties of metal NPs, either by mimetic-like activities or by the direct influence on antioxidative defense of the organism represented by antioxidant enzymes.

Literature data [57] suggest oxidative damage to lipids but no changes in activities of antioxidant enzymes after a short-term (24 h) exposure of fish to Ag NPs (average size 50 nm, dose 10-25 *μ*g Ag NPs/l of water). In another study [58], in liver homogenates, increased lipid peroxidation and elevated catalase and SOD activities were found after 14-day exposure of fish to metal oxide (Al_2_O_3_ and ZnO) NPs. We confirmed no alteration of the marker of oxidative damage to lipids—8-isoprostane in healthy HEK 293 T cells. On the contrary, 72-h incubation of cancer A549 cells with Au NPs increased its levels compared to 24-h incubation. However, compared to controls, the level of 8-isoprostane was decreased at both times of incubation. Interestingly, other cancer A375 cells behaved differently—8-isoprostane level increased after the treatment with 20 nm Au NPs for 24 h, as well as 72 h, except of the NPs concentration of 1.6 × 10^11^ pcs/mL, where it remained unchanged. Nevertheless, we can summarize the increase in lipid damage in both A549 and A375 cancer cells, which is in line with Alarifi et al.'s findings [43], who confirmed the elevation of lipid peroxidation in MCF-7 (breast cancer) cells. But unlike us, they determined the depletion of SOD and catalase activities in mentioned cancer cell line.

Sen et al. [9] also studied the effects of Au NPs (size of 55-65 nm, concentrations 25-400 *μ*g/mL, and 24 h incubation) on the oxidative stress of HepG2 cells characterized by activities of GPx, SOD, and catalase, as well as on the lipid peroxidation and protein oxidation. Compared to the control, they found no effects either on enzymatic activities or protein carbonyl level and lipid peroxidation characterized by malondialdehyde level. In contrast, our results indicate significantly increased oxidative damage to proteins (reflected by increased protein carbonyl levels) by Au NPs in A549 cells over time at all concentrations of NPs, but, inexplicable, also in the control. The similar increase was determined also in A375 cells, but not in healthy HEK 293 T cells.

Results of many studies on intracellular oxidative stress and its modification by the presence of metal NPs are contradictory. Moreover, many studies have found evidence of different behavior of metal oxide NPs and metal NPs. Likewise, different *in vitro* studies concluded inconsistent results on various cell lines. In addition, according to our results, there are also differences between NP interactions with healthy and cancer cells. All of these discrepancies in outcomes could be the goal of further research focused on the action of different types of metal NPs on diverse cell lines, tissues, or animal models.

## Figures and Tables

**Figure 1:** Viability of HEK 293 T (a), A375 (b), and A549 (c) cell lines during 24 h and 72 h treatment with 20 and 100 nm Au NPs. Concentration is given in pcs/ml. Results are expressed as mean ± SEM significance between control cells and cells incubated with NPs of a given size and concentration (∗*P* < 0.05, ∗∗*P* < 0.01).

**Table 1:** TEAC of HEK 293 T cells after 24 h and 72 h incubation with 20 nm and 100 nm Au NPs (pcs/mL).

Control or pcs/mL	24h TEAC (mmol of trolox/*μ*g proteins)		72h TEAC (mmol of trolox/*μ*g proteins)	
Control	0.032 (0.030–0.036)		0.038 (0.032–0.039)	
	20nm	100nm	20nm	100nm
1.6 × 10^7^		0.039 (0.032–0.070)		0.038 (0.035–0.039)
1.6 × 10^9^	0.025 (0.023–0.032)	0.030 (0.026–0.032)	0.038 (0.032–0.040)	0.033 (0.031–0.038)
1.6 × 10^11^	0.026 (0.025–0.048)		0.040 (0.030–0.044)	

Results are expressed as median (lower quartile–upper quartile).

**Table 2:** Concentration of 8-isoprostane in HEK 293 T cells after 24 h and 72 h incubation with 20 nm and 100 nm Au NPs (pcs/mL).

Control or pcs/mL	24 h∗ 8-isoprostane (pg/mL)		72 h 8-isoprostane (pg/mL)	
Control •	237.7 (232.4–246.4)		272.3∗ (265.7–287. 1)	
	20 nm	100 nm	20 nm	100 nm
1.6 × 10^7^		235.9 (234.1–242.4)		250.5∗ (249.5–250.5)
1.6 × 10^9^	235.0 (225.8–244.3)	241.4 (232.4–245.3)	248.41 (242.4–259.5)	268.3∗ (256–282.4)
1.6 × 10^11^	237.7 (230.7–246.4)		229.9••• (226.6–238.6)	

Results are expressed as median (lower quartile–upper quartile). ^•••^Significance between control cells and cells incubated with NPs of a given size and concentration (*P* < 0.001). ∗Significance over time (between 24h and 72h) in cells incubated with NPs of a given size and concentration (*P* < 0.05).

**Table 3:** Concentration of protein carbonyls in HEK 293 T cells after 24 h and 72 h incubation with 20 nm and 100 nm Au NPs (pcs/mL).

Control or pcs/mL	24 h∗ Protein carbonyls (nmol/mg proteins)		72 h Protein carbonyls (nmol/mg proteins)	
Control •	1059 (1052.5–1065.8)		1540.9∗∗ (1531–1545.9)	
	20 nm	100 nm	20 nm	100 nm
1.6×10^7^		859.9 (851.8–863.9)		1161.1 (1149.2–1176.1)
1.6×10^9^ +	1098.8 (1090.7–1104.5)	762.2• (759.1–765.9)	1322.8 (1307.8–1342.3)	924.2•• (918.5–937.0)
1.6×10^11^	769.5+ (768.8–776.7)		1254.0 (1248.0–1263.0)	

Results are expressed as median (lower quartile–upper quartile). ^•^, ^••^Significance between control cells and cells incubated with NPs of a given size and concentration (^•^*P* < 0.05, ^••^*P* < 0.01). ∗∗Significance over time (between 24 h and 72 h) in cells incubated without/with NPs of a given size and concentration (*P* < 0.01). +: Significance between cells incubated with 20 nm NPs at the concentration of 1.6 × 10^9^ pcs/mL and cells incubated with 20 nm NPs of different concentration (*P* < 0.05).

**Table 4:** SOD activity in HEK 293 T cells after 24 h and 72 h incubation with 20 nm and 100 nm Au NPs (pcs/mL).

Controls or pcs/mL	24 h∗ SOD activity (inhibition rate percent)		72 h SOD activity (inhibition rate percent)	
Control	69.36 (66.52–71.55)		72.867 (70.9–75.71)	
	20 nm	100 nm	20 nm	100 nm
1.6 × 10^7^		71.99 (66.30–73.52)		67.62 (63.02–74.18)
1.6 × 10^9^	66.08 (66.08–73.09)	76.15 (75.06–77.46)	75.49 (61.05–79.43)	66.30∗ (66.08–73.3)
1.6 × 10^11^	64.99 (61.05–72.21)		69.80 (68.05–69.8)	

Results are expressed as median (lower quartile–upper quartile). ∗Significance over time (between 24 h and 72 h) in cells incubated with NPs of a given size and concentration (*P* < 0.05).

**Table 5:** GPx activity of HEK-293 T cells after 24 h and 72 h incubation with 20 nm and 100 nm Au NPs (pcs/mL).

Control or pcs/mL	24 h GPx activity (U/mg proteins)		72 h GPx activity (U/mg proteins)	
Control	0.198 (0.169–0.254)		0.254 (0.198–0.282)	
	20 nm	100 nm	20 nm	100 nm
1.6 × 10^7^		0.226 (0.212–0.226)		0.254 (0.254–0.282)
1.6 × 10^9^	0.240 (0.183 – 0.282)	0.212 (0.141–0.282)	0.212 (0.169–0.282)	0.212 (0.198–0.226)
1.6 × 10^11^	0.226 (0.155 – 0.240)		0.169 (0.155–0.226)	

Results are expressed as the median (lower quartile–upper quartile).

**Table 6:** Catalase activity of HEK 293 T cells after 24 h or 72 h incubation with 20 nm and 100 nm Au NPs (pcs/mL).

Control or pcs/mL	24 h∗ Catalase activity (U/mg proteins)		72 h Catalase activity (U/mg proteins)	
Control •	2.00 (1.31–2.51)		2.7 (2.00 – 3.53)	
	20 nm	100 nm	20 nm	100 nm
1.6 × 10^7^		3.91• (3.72–10.25)		3.78 (3.40–3.84)
1.6 × 10^9^	2.83 (2.77–2.89)	3.21 (2.39–3.53)	3.84∗ (3.53–3.84)	1.497 (1.18–1.69)
1.6 × 10^11^	5.43• (5.30–6.51)		3.97 (3.53–4.73)	

Results are expressed as median (lower quartile–upper quartile). ^•^Significance between control cells and cells incubated with NPs of a given size and concentration (*P* < 0.05). ∗Significance over time (between 24h and 72h) in cells incubated with NPs of a given size and concentration (*P* < 0.05).

**Table 7:** TEAC of A375 cells after 24 h and 72 h incubation with 20 nm and 100 nm Au NPs (pcs/mL).

Control or pcs/mL	24 h∗ TEAC (mmol of trolox/*μ*g proteins)		72 h TEAC (mmol of trolox/*μ*g proteins)	
Control •	0.049 (0.049–0.049)		0.058 (0.058–0.060)	
	20 nm	100 nm	20 nm	100 nm
1.6×10^7^		0.053 (0.052–0.053)		0.045•¥¥¥ (0.043–0.047)
1.6×10^9^ ¥	0.042 (0.041–0.043)	0.051 (0.044–0.053)	0.057∗∗ (0.050–0.060)	0.066∗ (0.060–0.069)
1.6×10^11^	0.050 (0.048–0.065)		0.050 (0.049–0.055)	

Results are expressed as median (lower quartile–upper quartile). ^•^Significance between control cells and cells incubated with NPs of a given size and concentration (^•^*P* < 0.05). ∗, ∗∗Significance over time (between 24 h and 72 h) in cells incubated with NPs of a given size and concentration (∗*P* < 0.05, ∗∗*P* < 0.01). ¥¥¥: Significance between cells incubated with 100 nm NPs with the concentration of 1.6 × 10^9^ pcs/mL and cells incubated with 100 nm NPs of a given concentration (*P* < 0.001).

**Table 8:** Concentration of 8-isoprostane in A375 cells after 24 h and 72 h incubation with 20 nm and 100 nm Au NPs (pcs/mL).

Control or pcs/mL	24 h∗ 8-isoprostane (pg/mL)		72 h 8-isoprostane (pg/mL)	
Control •	238.6 (226.63–246.35)		238.6 (230.7–242.38)	
	20 nm	100 nm	20 nm	100 nm
1.6 × 10^7^		252.68 (243.36–264.4)		245.34 (236.78–256.03)
1.6 × 10^9^+	239.53 (226.63–244.34)	240.47 (227.42–248.41)	276.47•∗ (257.18–283.92)	246.35 (239.53–257.18)
1.6 × 10^11^	263.16•+ (250.52–276.47)		232.39 (225.06–234.11)	

Results are expressed as median (lower quartile–upper quartile). ^•^Significance between control cells and cells incubated with NPs of a given size and concentration (^•^*P* < 0.05). ∗Significance over time (between 24 h and 72 h) in cells incubated with NPs of a given size and concentration (∗*P* < 0.05). +: Significance between cells incubated with 20 nm NPs at the concentrations of 1.6 × 10^9^ pcs/mL and 1.6 × 10^11^ pcs/mL (+*P* < 0.05).

**Table 9:** Concentration of protein carbonyls in A375 cells after 24 h and 72 h incubation with 20 nm and 100 nm Au NPs (pcs/mL).

Control or pcs/mL	24 h∗ Protein carbonyls (nmol/mg proteins)		72 h Protein carbonyls (nmol/mg proteins)	
Control •	201.4 (197.1-205.7)		1346.7∗∗ (1331.1-1365.8)	
	20 nm	100 nm	20 nm	100 nm
1.6 × 10^7^		1006.6••• (1000.9-1020.8)		1292.7∗∗ (1277-1303.7)
1.6 × 10^9^	739.3 (732.8-746.0)	1036.4••• (1023.9-1040.2)	1750.1∗ (1742.2-1756.5)	1329.8 (1318.4-1344)
1.6 × 10^11^	462.3 (454.0-470.6)		1358.0∗ (1343.5-1362.4)	

Results are expressed as median (lower quartile–upper quartile). ^•••^Significance between control cells and cells incubated with NPs of a given size and concentration (^•••^*P* < 0.001). ∗, ∗∗Significance over time (between 24 h and 72 h) in cells incubated with NPs of a given size and concentration (∗*P* < 0.05, ∗∗*P* < 0.01).

**Table 10:** SOD activity of A375 cells after 24 h and 72 h incubation with 20 nm and 100 nm Au NPs (pcs/mL).

Control or pcs/mL	24 h∗ SOD activity (inhibition rate percent)		72 h SOD activity (inhibition rate percent)	
Control	50.65 (44.89–55.07)		49.98 (48.88–57.95)	
	20 nm	100 nm	20 nm	100 nm
1.6 × 10^7^		45.55 (22.32–50.42)		46.11 (25.86–66.36)
1.6 × 10^9^	30.06 (21.87–46.88)	47.77 (40.24–63.26)	56.62∗ (56.18–58.39)	46.88 (46.22–51.31)
1.6 × 10^11^	56.84 (39.36–64.81)		54.41 (54.41–54.41)	

Results are expressed as median (lower quartile–upper quartile).

∗Significance over time (between 24 h and 72 h) in cells incubated with NPs of a given size and concentration (∗*P* < 0.05).

**Table 11:** GPx activity of A375 cells after 24 h and 72 h incubation with 20 nm and 100 nm Au NPs (pcs/mL).

Control or pcs/mL	24 h GPx activity (U/mg proteins)		72 h GPx activity (U/mg proteins)	
Control	0.198 (0.155–0.282)		0.254 (0.141 – 0.381)	
	20 nm	100 nm	20 nm	100 nm
1.6 × 10^7^		0.226 (0.2120.325)		0.282 (0.254–0.381)
1.6 × 10^9^	0.226 (0.198–0.296)	0.212 (0.183–0.296)	0.282 (0.282–0.367)	0.268 (0.155–0.367)
1.6 × 10^11^	0.240 (0.183–0.353)		0.240 (0.198–0.296)	

Results are expressed as median (lower quartile–upper quartile).

**Table 12:** Catalase activity of A375 cells after 24 h and 72 h incubation with 20 nm and 100 nm Au NPs (pcs/mL).

Control or pcs/mL	24 h∗ Catalase activity (U/mg proteins)		72 h Catalase activity (U/mg proteins)	
Control •	5.37 (5.37–5.75)		2.2∗∗ (2.2–2.45)	
	20 nm	100 nm	20 nm	100 nm
1.6 × 10^7^		3.27• (2.58–3.27)		4.669 (4.16–5.05)
1.6 × 10^9^+	11.08 (11.08–11.46)	5.05 (0.67–5.05)	4.1∗ (3.78–4.29)	11.58••• (11.33–11.77)
1.6 × 10^11^	0.61••+++ (0.61–1.05)		2.7∗ (2.45–2.83)	

Results are expressed as median (lower quartile–upper quartile). ^•^,^••^,^•••^Significance between control cells and cells incubated with NPs of a given size and concentration (^•^*P* < 0.05, ^••^*P* < 0.01, ^•••^*P* < 0.001). ∗Significance over time (between 24 h and 72 h) in cells incubated with NPs of a given size and concentration (∗*P* < 0.05). +++: Significance between cells incubated with 20 nm NPs at concentrations of 1.6 × 10^9^ pcs/mL and 1.6 × 10^11^ pcs/mL (+++*P* < 0.001).

**Table 13:** TEAC of A549 cells after 24 h and 72 h incubation with 20 nm and 100 nm Au NPs (pcs/mL).

Controls or pcs/mL	24 h∗ TEAC (mmol of trolox/*μ*g proteins)		72 h TEAC (mmol of trolox/*μ*g proteins)	
Control •	0.041 (0.040-0.044)		0.056∗ (0.056-0.059)	
	20 nm	100 nm	20 nm	100 nm
1.6 × 10^7^		0.063•¥¥¥ (0.059-0.063)		0.040•••∗¥ (0.032-0.040)
1.6 × 10^9^ + ¥	0.040 (0.036-0.042)	0.033 (0.029-0.036)	0.046 (0.043-0.049)	0.054∗ (0.047-0.054)
1.6 × 10^11^	**0.054**•**+** (0.053-0.059)		0.040••∗ (0.034-0.042)	

Results are expressed as median (lower quartile–upper quartile). ^•^,^••^,^•••^Significance between control cells and cells incubated with NPs of a given size and concentration (^•^*P* < 0.05, ^••^*P* < 0.01, ^•••^*P* < 0.001). ∗Significance over time (between 24 h and 72 h) in cells incubated with NPs of a given size and concentration (∗*P* < 0.05). +: Significance between cells incubated with 20 nm NPs at concentrations of 1.6 × 10^9^ pcs/mL and 1.6 × 10^11^ pcs/mL (+*P* < 0.05). ¥, ¥¥¥: Significance between cells incubated with 100 nm NPs at concentration of 1.6 × 10^9^ pcs/mL and 1.6 × 10^7^ pcs/mL (¥*P* < 0.05, ¥¥¥*P* < 0.001).

**Table 14:** Concentration of 8-isoprostane in A549 cells after 24 h and 72 h incubation with 20 nm and 100 nm Au NPs (pcs/mL).

Control or pcs/mL	24 h∗ 8-isoprostane (pg/mL)		72 h 8-isoprostane (pg/mL)	
Control•	295.43 (288.69-314.6)		290.330 (279.376-302.673)	
	20 nm	100 nm	20 nm	100 nm
1.6×10^7^		265.67 (258.35-276.47)		323.37∗∗¥¥ (297.2-343.35)
1.6×10^9^ ¥	248.41•• (242.38-257.18)	277.91 (273.64-293.70)	270.91 (266.95-285.48)	259.52• (253.79-265.67)
1.6×10^11^	258.35• (256.03-266.95)		302.67∗∗ (288.69-316.72)	

Results are expressed as median (lower quartile–upper quartile). ^•^,^••^Significance between control cells and cells incubated with NPs of a given size and concentration (^•^*P* < 0.05, ^••^*P* < 0.01). ∗∗Significance over time (between 24 h and 72 h) in cells incubated with NPs of a given size and concentration (∗∗*P* < 0.01). ¥¥: Significance between cells incubated with 100 nm NPs at the concentrations of 1.6 × 10^9^ pcs/mL and 1.6 × 10^7^ pcs/mL (¥¥*P* < 0.01).

**Table 15:** Concentration of protein carbonyls in A549 cells after 24 h and 72 h incubation with 20 nm and 100 nm Au NPs (pcs/mL).

Control or pcs/mL	24 h∗ Protein carbonyls (nmol/mg proteins)		72 h Protein carbonyls (nmol/mg proteins)	
Control•	74.93 (70.24-82.42)		384.535∗∗ (374.036-393.722)	
	20 nm	100 nm	20 nm	100 nm
1.6 × 10^7^		72 (2.45 - 77.72)		111.92•∗¥¥ (101.48-116.4)
1.6 × 10^9^ + ¥	56.83 (51.58-62.95)	75.83 (69.26-81.66)	243.45∗∗ (232.86-256.68)	402.31∗ (397.03-412.87)
1.6 × 10^11^	100.14+++ (95.22-106.71)		256.17∗∗ (251.42-268.02)	

Results are expressed as median (lower quartile–upper quartile). ^•^Significance between control cells and cells incubated with NPs of a given size and concentration (^•^*P* < 0.05). ∗,∗∗Significance over time (between 24 h and 72 h) in cells incubated with NPs of a given size and concentration (∗*P* < 0.05, ∗∗*P* < 0.01). +++: Significance between cells incubated with 20 nm NPs at concentrations of 1.6 × 10^9^ pcs/mL and 1.6 × 10^11^ pcs/mL (+++*P* < 0.001). ¥¥: Significance between cells incubated with 100 nm NPs at concentrations of 1.6 × 10^7^ pcs/mL and 1.6 × 10^9^ pcs/mL (¥¥*P* < 0.01).

**Table 16:** SOD activity of A549 cells after 24 h and 72 h incubation with 20 nm and 100 nm Au NPs (pcs/mL).

Control or pcs/mL	24 h∗ SOD activity (inhibition rate percent)		72 h SOD activity (inhibition rate percent)	
Control •	59.06 (56.82-64.88)		69.8 (67.56-75.17)	
	20 nm	100 nm	20 nm	100 nm
1.6 × 10^7^		58.17 (54.59-58.39)		68.01 (60.85-69.8)
1.6 × 10^9^	61.75 (53.02-65.77)	63.31 (57.05-71.14)	73.83∗ (73.60-100.00)	64.43 (60.18-69.58)
1.6 × 10^11^	64.21 (62.64-75.62)		68.23 (56.82-70.92)	

Results are expressed as median (lower quartile–upper quartile). ∗Significance over time (between 24 h and 72 h) in cells incubated with NPs of a given size and concentration (∗*P* < 0.05).

**Table 17:** GPx activity of A549 cells after 24 h and 72 h incubation with 20 nm and 100 nm Au NPs (pcs/mL).

Control or pcs/mL	24 h∗ GPx activity (U/mg proteins)		72 h GPx activity (U/mg proteins)	
Control	0.212 (0.198-0.254)		0.155∗ (0.028-0.169)	
	20 nm	100 nm	20 nm	100 nm
1.6 × 10^7^		0.169 (0.169 - 0.198)		0.226 (0.127-0.254)
1.6 × 10^9^	0.183 (0.155-0.198)	0.183 (0.141-0.226)	0.141 (0.028-0.183)	0.169 (0.169-0.212)
1.6 × 10^11^	0.198 (0.141-0.212)		0.141 (0.014-0.198)	

Results are expressed as median (lower quartile–upper quartile). ∗Significance over time (between 24 h and 72 h) in cells incubated with NPs of a given size and concentration (∗*P* < 0.05).

**Table 18:** Catalase activity of A549 cells after 24 h and 72 h incubation with 20 nm and 100 nm Au NPs (pcs/mL).

Control or pcs/mL	24 h∗ Catalase activity (U/mg proteins)		72 h Catalase activity (U/mg proteins)	
Control•	2.07 (1.94-2.2)		0.74 (0.67-0.8)	
	20 nm	100 nm	20 nm	100 nm
1.6 × 10^7^		1.94 (1.56-2.13)		3.46¥ (3.27-3.65)
1.6 × 10^9^ + ¥	1.18 (0.8-1.43)	3.02 (2.96-3.53)	1.751 (1.37-2.96)	8.09•••∗∗ (7.46-8.45)
1.6 × 10^11^	5.18+++ (4.99-5.3)		6.89•••++ (6.38-7.21)	

Results are expressed as median (lower quartile–upper quartile). ^•••^Significance between control cells and cells incubated with NPs of a given size and concentration (^•••^*P* < 0.001). ∗∗Significance over time (between 24 h and 72 h) in cells incubated with NPs of a given size and concentration (∗∗*P* < 0.01). ++, +++: Significance between cells incubated with 20 nm NPs at concentrations of 1.6 × 10^9^ pcs/mL and 1.6 × 10^11^ pcs/mL (++*P* < 0.01, +++*P* < 0.001). ¥: significance between cells incubated with 100 nm NPs at concentrations of 1.6 × 10^9^ pcs/mL and 1.6 × 10^7^ pcs/mL (¥*P* < 0.01).

## Data Availability

Underlying data will be sent on request.

## References

[1] Borm P. J., Robins D., Haubold S. (2006). The potential risks of nanomaterials: a review carried out for ECETOC. *Particle and Fibre Toxicology*.

[2] Stapleton P., Turkiewitz T. (2014). Vascular distribution of nanomaterials. *Wiley Interdisciplinary Reviews. Nanomedicine and Nanobiotechnology*.

[3] Kang S., Kim Y., Chung H. (2008). Titanium dioxide nanoparticles trigger p 53-mediated damage response in peripheral blood lymphocytes. *Environmental and Molecular Mutagenesis*.

[4] Gurunathan S., Jeyaraj M., Kang M.-H., Kim J.-H. (2019). Tangeretin-assisted platinum nanoparticles enhance the apoptotic properties of doxorubicin: combination therapy for osteosarcoma treatment. *Nanomaterials*.

[5] Foster H., Ditta I., Varghese S., Steele A. (2011). Photocatalytic disinfection using titanium dioxide: spectrum and mechanism of antimicrobial activity. *Applied Microbiology and Biotechnology*.

[6] Lee J., Kwon E.-S., Kim D.-W., Cha J., Roe J.-H. (2002). Regulation and the role of Cu, Zn-containing superoxide dismutase in cell cycle progression of Schizosaccharomyces pombe. *Biomedical and Biophysical Research Communitacions*.

[7] Yamada K., Nakagawa C., Mutoh N. (1999). Schizosaccharomyces pombe homologue of glutathione peroxidase, which does not contain selenocysteine, is induced by several stresses and works as an antioxidant. *Yeast*.

[8] Mody V., Siwale R., Singh A., Mody H. (2010). Introduction to metallic nanoparticles. *Journal of Pharmacy and bioallied sciences*.

[9] Sen G., Ozkemahli G., Shahbazi R., Erkekoglu P., Ulubayram K., Kocer-Gumusel B. (2020). The effects of polymer coating of gold nanoparticles on oxidative stress and DNA damage. *International Journal of Toxicology*.

[10] Giljohan D., Seferos D., Daniel W., Massich M., Patel P., Mirkin C. (2010). Gold nanoparticles for biology and medicine. *Spherical Nucleic Acids*.

[11] El-Sayed I., Huang X., El-Sayed M. (2005). Surface plasmon resonance scattering and absorption of anti-EGFR antibody conjugated gold nanoparticles in cancer diagnostics: applications in oral cancer. *Nano Letters*.

[12] Habibullah G., Viktorova J., Ruml T. (2021). Current strategies for noble metal nanoparticle synthesis. *Nanoscale Research Letters*.

[13] Mody V., Nounou M., Bikram M. (2009). Novel nanomedicine-based MRI contrast agents for gynecological malignancies. *Advanced Drug Delivery Reviews*.

[14] Guerrero-Florez V., Mendez-Sanchez S., Patrón-Soberano O., Rodrígez-González V., Blach D., Martinez F. (2020). Gold nanoparticle-mediated generation of reactive oxygen species during plasmonic photothermal therapy: a comparative study for different particle sizes, shapes, and surface conjugations. *Journal of Materials Chemistry B*.

[15] Okkeh M., Bloise N., Restivo E., De Vita L., Pallavicini P., Visai L. (2021). Gold nanoparticles: can they be the next magic bullet for multidrug-resistant bacteria?. *Nanomaterials*.

[16] Ahamed M., Akhtar M., Alaizeri Z., Alhadlaq H. (2020). TiO2 nanoparticles potentiated the cytotoxicity, oxidative stress and apoptosis response of cadmium in two different human cells. *Environmental Science and Pollution Reasearch*.

[17] Akter M., Sikder M., Rahman M. (2018). A systematic review on silver nanoparticles-induced cytotoxicity: physicochemical properties and perspectives. *Journal of Advanced Research*.

[18] Rajoria S., Rani S., Chaudhari D., Jain S., Gupta U. (2019). Glycine-poly-L-lactic acid copolymeric nanoparticles for the efficient delivery of bortezomib. *Pharmaceutical Research*.

[19] Yu Z., Li Q., Wang J. (2020). Reactive oxygen species-related nanoparticle toxicity in the biomedical field. *Nanoscale Research Letters*.

[20] Ahamed M., Akhtar M., Khan M., Alrokayan S., Alhadlaq H. (2019). Oxidative stress mediated cytotoxicity and apoptosis response of bismuth oxide (Bi2O3) nanoparticles in human breast cancer (MCF-7) cells. *Chemosphere*.

[21] Stater E., Sonay A., Hart C., Grimm J. (2021). The ancillary effects of nanoparticles and their implications for nanomedicine. *Nature Nanotechnology*.

[22] Wolfram J., Zhu M., Yang Y. (2015). Safety of nanoparticles in medicine. *Current Drugs Targets*.

[23] Ji L., Yeo D. (2021). Oxidative stress: an evolving definition. *Faculty Reviews*.

[24] Sies H. (2020). Oxidative stress: concept and some practical aspects. *Antioxidants*.

[25] Haliwell B., Gutteridge J. (2015). *Free radicals in biology and medicine*.

[26] Droge W. (2002). Free radicals in the physiological control of cell function. *Physiological Reviews*.

[27] Pizzino G., Irrera N., Cucinotta M. (2017). Oxidative stress: harms and benefits for human health. *Oxidative Medicine and Cellular Longevity*.

[28] Taysi S., Tascan A., Ugur M., Demir M. (2019). Radicals, oxidative/nitrosative stress and preeclampsia. *Mini Reviews in Medicinal Chemistry*.

[29] Ahamed M., Akhtar M., Khan M., Alhadlaq H. (2021). Co-exposure of Bi2O3 nanoparticles and bezo[a]pyrene-enhanced in vitro cytotoxicity of mouse spermatogonia cells. *Environmental Science and Pollution Research*.

[30] Li Y., Quin T., Ingle T. (2017). Differential genotoxicity mechanisms of silver nanoparticles and silver ions. *Archives of Toxicology*.

[31] Ahmed B., Hashmi A., Khan M., Musarrat J. (2018). ROS mediated destruction of cell membrane, growth and biofilms of human bacterial pathogens by stable metallic AgNPs functionalized from bell pepper extract and quercetin. *Advanced Powder Technology*.

[32] Čapek J., Roušek T. (2021). Detection of oxidative stress induced by nanomaterials in cells-the roles of reactive oxygen species and glutathione. *Molecules*.

[33] Ge D., Du Q., Ran B. (2019). The neurotoxicity induced by engineered nanomaterials. *International Journal of Nanomedicine*.

[34] Ahamed M., Akhtar M., Raja M. (2011). ZnO nanorod-induced apoptosis in human alveolar adenocarcinoma cells via p53, survivin and bax/bcl-2 pathways: role of oxidative stress. *Nanomedicine*.

[35] Horie M., Tabei Y. (2021). Role of oxidative stress in nanoparticles toxicity. *Free Radical Research*.

[36] Mauricio M. D., Guerra-Ojeda S., Marchio P. (2018). Nanoparticles in medicine: a focus on vascular oxidative stress. *Oxidative Medicine and Cellular Longevity*.

[37] Mosman T. (1983). Rapid colorimetric assay for cellular growth and survival: application to proliferation and cytotoxicity assays. *Journal of Immunological Methods*.

[38] Re R., Pellegrini N., Proteggente A., Pannala A., Yang M., Rice-Evans C. (1999). Antioxidant activity applying an improved ABTS radical cation decolorization assay. *Free Radical Biology and Medicine*.

[39] Dhawan A., Sharma V. (2010). Toxicity assessment of nanomaterials: methods and challenges. *Analytical and Bioanalytical Chemistry*.

[40] Paciorek P., Zuberek M., Grzelak A. (2020). Products of lipid peroxidation as a factor in the toxic effect of silver nanoparticles. *Materials*.

[41] Sahu S., Hayes W. (2017). Toxicity of nanomaterials found in human environment: a literature review. *Toxicology Research and Application*.

[42] Zuberek M., Grzelak A. (2018). Nanoparticles-caused oxidative imbalance. In Q. Saquib, M. Faisal, A. Al-Khedhairy, & a. Alatar, cellular and molecular toxicology of nanoparticles. *Advances in Experimental Medicine and Biology*.

[43] Alarifi S., Ali D., Alkahtani S., Alhader M. (2014). Iron oxide nanoparticles induce oxidative stress, DNA damage, and caspase activation in the human breast cancer cell line. *Biological Trace Element Research*.

[44] Sooklert K., Chattong S., Manotham K. (2016). Cytoprotective effect of glutaraldehyde erythropoietin on HEK293 kidney cells after silver nanoparticle exposure. *International Journal of Nanomedicine*.

[45] Sims C., Hanna S., Heller D. (2017). Redox-active nanomaterials for nanomedicine applications. *Nanoscale*.

[46] Cao G.-J., Jiang X., Zhang H., Zheng J., Croley T., Yin J.-J. (2017). Exploring the activities of ruthenium nanomaterials as reactive oxygen species scavengers. *Journal of Environmental Science and Health*.

[47] Chen J., Wang Q., Huang L. (2018). Prussian blue with intrinsic heme-like structure as peroxidase mimic. *Nano Research*.

[48] Li C.-W., Li L.-L., Zhang J.-X., Lu W.-L. (2020). Antioxidant nanotherapies for the treatment of inflammatory diseases. *Frontiers in Bioengineering and Biotechnology*.

[49] Keshari A., Srivastava R., Singh P., Yadav P., Yadav V., Nath G. (2020). Antioxidant and antibacterila activity of silver nanoparticles synthesized by Cestrum nocturnum. *Journal of Ayurveda and Integrative Medicine*.

[50] Annu M., Ahmed S., Kaur G., Sharma P., Singh S., Ikram S. (2018). Evaluation of the antioxidant, antibacterial and anticancer (lung cancer cell line A549) activity ofPunica granatummediated silver nanoparticles. *Toxicology Research*.

[51] Xia T., Kovochich M., Liong M. (2008). Comparison of the mechanism of toxicity of zinc oxide and cerium oxide nanoparticles based on dissolution and oxidative stress properties. *ACS Nano*.

[52] Srinivas A., Rao P., Selvam G., Murthy P., Reddy P. (2011). Acute inhalation toxicity of cerium oxide nanoparticles in rats. *Toxicology Letters*.

[53] Siddiqi N. (2014). Effect of gold nanoparticles on superoxide dismutase and indoleamine 2, 3-dioxygenase in various rat tissues. *Indian Journal of Biochemistry & Biophysics*.

[54] Lee J., Yoon S., Lo M., Wu H., Lee S., Moon B. (2015). Intrinsic polyphenol oxidase-like activity of gold@platinum nanoparticles. *RSC Advances*.

[55] Canli E., Canli M. (2020). Effects of aluminum, copper and titanium nanoparticles on the liver antioxidant enzymes of the Nile fish (Oreochromis niloticus). *Energy Reports*.

[56] Ismail N., Lee J., Yusof F. (2022). Platinum nanoparticles: the potential antioxidant in the human lung cancer cells. *Antioidants*.

[57] Bacchetta C., Ale A., Simoniello M. (2017). Genotoxicity and oxidative stress in fish after a short-term exposure to silver nanoparticles. *Ecological Indicators*.

[58] Benavides M., Fernández-Lodeiro J., Coelho P., Lodeiro C., Diniz M. (2016). Single and combined effects of aluminum (Al2O3) and zinc (ZnO) oxide nanoparticles in a freshwater fish, Carassius auratus. *Environmental Science and Pollution Research*.

